# Wogonin reversed resistant human myelogenous leukemia cells via inhibiting Nrf2 signaling by Stat3/NF-κB inactivation

**DOI:** 10.1038/srep39950

**Published:** 2017-02-02

**Authors:** Xuefen Xu, Xiaobo Zhang, Yi Zhang, Lin Yang, Yicheng Liu, Shaoliang Huang, Lu Lu, Lingyi Kong, Zhiyu Li, Qinglong Guo, Li Zhao

**Affiliations:** 1 State Key Laboratory of Natural Medicines, Jiangsu Key Laboratory of Carcinogenesis and Intervention, China Pharmaceutical University, 24 Tongjiaxiang, Nanjing, 210009, People’s Republic of China; 2 State Key Laboratory of Natural Medicines, Department of Natural Medicinal Chemistry, China Pharmaceutical University, 24 Tongjiaxiang, Nanjing, 210009, People’s Republic of China

## Abstract

Constitutive NF-E2-related factor 2 (Nrf2, NFE2L2) activation has been recently reported to play a pivotal role in enhancing cell survival and resistance to anticancer drugs in many tumors. Wogonin had strong reversal potency via reduction of *Nrf2* mRNA in Adriamycin (ADR)-induced resistant human chronic myelogenous leukemia (CML) K562/A02, but the mechanism of reduction of *Nrf2* mRNA was still unclear. In this study, we aimed to delineate the mechanism by which Wogonin suppressed transcription of *Nrf2* in resistant CML cells and further evaluate the reversal effects of Wogonin on the established animal models. Data indicated that Wogonin suppressed transcription of *Nrf2* by NF-κB inactivation. Wogonin inhibited the binding of p65 to Nrf2 by suppression of the κB-binding activity. Further research revealed the κB2 site was responsible for the decreased Nrf2 by Wogonin in resistant K562 cells. Furthermore, reduction of pY705-Stat3 was involved in inhibition of the binding of p65 to Nrf2 by Wogonin. *In vivo*, Wogonin potentiated the inhibitory effect of ADR on leukemia development by suppressing pY705-Stat3 and Nrf2 signaling. In summary, these results demonstrated Wogonin could combat chemoresistance effectively through inhibiting Nrf2 via Stat3/NF-κB signaling, and supported that Wogonin can be developed into an efficient natural sensitizer for resistant human myelogenous leukemia.

The most significant cause of treatment failure in CML is the multidrug resistance (MDR) of leukemia cells^1^. BCR-ABL specific tyrosine kinase inhibitors (TKIs), such as Imatinib (IM), Nilotinib and Dasatinib, have improved the 10-years survival time in 80% CML patients^2^. However, BCR/ABL^+^ disease remains detectable in essentially all patients with chronic-phase CML, and cessation of drug treatment leads to disease recurrence in most CML patients^3^. This may be due to an inherent inhibitor resistance of quiescent progenitors and BCR/ABL overexpression^4^. Other mechanisms include BCR/ABL kinase mutations^5^, increased expression of the drug transporter ABCB1^6^, elevated levels of granulocyte-macrophage colony-stimulating factor (GM-CSF)^7^, or TP53 inactivation^8^. However, additional aberrations of signal transduction pathways may be required to cause a fully drug-resistant phenotype^9^.

Recently, a number of potential anticancer therapies have emerged that are targeted to specific signaling pathways or cellular processes resulting in apoptosis^10^. Many potential anticancer therapies are being evaluated, but their efficacies, roles, and modes of action as either single agents or combined with other drugs are required to be further clarified. One pathway being targeted was the ubiquitin-proteasome system that regulated protein turnover and many cellular processes, including gene regulation, cell cycle, and oxidative stress responses. Nrf2 and NF-κB were 2 transcription factors regulated by the ubiquitin-proteasome system^11^,^12^. Both NF-κB and Nrf2 pathways activated many survival signaling pathways known to play pivotal roles in protecting cancer cells from anticancer therapies cytotoxicity^13^,^14^. NF-κB is a family of transcription factors that share homology to the retroviral oncoprotein v-Rel. Resistant cancer cells showed aberrant or constitutive NF-κB activation, which initiated anti-apoptotic protein expression, augmented proinflammatory cytokine secretion and contributed to MDR^15^. Emerging evidence supported a functional interplay between Nrf2 and NF-κB signaling pathways, which contributed to generate additional complexity to the regulation of cell behavior. For example, it has been reported that Nrf2-deficient mouse embryonic fibroblasts exhibited greater activation of NF-κB in response to LPS stimulus^16^, and Nrf2^−/−^ mice were more susceptible to brain injury-induced cerebral NF-κB activation including inflammatory cytokine TNFα, IL-1β, and IL-6 production^17^. Conversely, NF-κB signaling could directly repress Nrf2 through competing transcription co-activator CBP and recruiting HDAC3 to cause local hypoacetylation^18^. As recently shown in human AML high Nrf2 was not linked to mutations in Nrf2, but was in fact the result of an aberrant or constitutive Nrf2 activation by NF-κB pathway^19^.

Nrf2 is one of the cancer cell survival pathways that plays a pivotal role in protecting cancer cells from apoptosis^20^. Nrf2 rapidly changes the sensitivity of the cells environment to oxidants and electrophiles by stimulating the transcriptional activation of over a hundred cytoprotective and detoxification genes, including antioxidants ferritin, glutathione-S-reductase (GSR), and glutamyl cysteine ligase modulator (GCLM) and catalytic (GCLC), phase I drug oxidation enzyme NAD (P) H:quinone oxidoreductase 1 (NQO1), and cytoprotective enzyme heme oxygenase-1 (HO-1) genes^21^. With respect to HO-1, other transcription factors including NF-κB and AP-1 are also involved in its expression^22^. Under normal physiologic conditions, the inhibitor of Nrf2, Keap1, mediates the ubiquitin-26S proteasome-mediated turnover of Nrf2. Exposure to oxidative and electrophilic stresses, such as reactive oxygen species (ROS) or chemotherapeutic agents, impairs Keap1-mediated proteasomal degradation of Nrf2, causing Nrf2 activation and translocation to the nucleus^23^. Then Nrf2 forms a complex with Maf proteins, which bind to the antioxidant response element (ARE) to mediate transcription of Nrf2-inducible genes^24^. Therefore, under normal cellular conditions Nrf2 is anticancerous because of upregulation of cytoprotective and detoxification proteins that protect cells from electrophilic/oxidative damage. Paradoxically, however, these cytoprotective and detoxification proteins that provide protection from cancer initiation enhance the resistance of cancer cells to chemotherapeutic drugs, and in this context Nrf2 is rapidly attracting a protumoral identity^25^,^26^.

Investigations have shown that constitutively high level of Nrf2 promotes cancer cell survival and is responsible for chemoresistance^27^. Inversely, downregulation of the Nrf2-dependent response by overexpression of Keap1 or knockdown of *Nrf2* increased sensitivity of anticancer drugs^28^. A variety of natural and synthetic chemicals have been identified as potent inhibitors of Nrf2, and such compounds may be used to increase the efficacy of anticancer drugs. Flavonoids, a diverse family of natural polyphenolic compounds commonly occurring in plants, was able to sensitize cancer cells to anticancer drugs^29^. Recently, Kweon *et al*.^30^ reported that epigallocatechin 3-gallate (EGCG), the major polyphenol found in green tea, suppressed HO-1 expression by inactivation of Nrf2 in non-small-cell lung cancer (NSCLC) A549 cells. Brusatol inhibited the Nrf2 signaling pathway and enhanced sensitivity of a broad spectrum of cancer cells and A549 xenografts to cisplatin^31^. Luteolin (30,40,5,7-tetrahydroxyflavone), a flavonoid found in high concentrations in celery, green pepper, parsley, perilla leaf, and chamomile tea, inhibited the Nrf2/ARE signaling, reduced cellular GSH level and sensitized A549 cells to therapeutic drugs^32^. The universal presence of flavonoids in dietary plants and their anticancer properties prompted us to determine whether other flavonoids can antagonize the Nrf2/ARE signaling pathway more potently.

Wogonin (5,7-dihydroxy-8-methoxyflavone), one of the major flavonoids isolated from the root of Scutellaria baicalensis Georgi, is the most promising anticancer candidate^33^ due to its antiproliferating, apoptosis-inducing, angiogenesis-inhibiting, cell migration-inhibiting and differentiation-inducing activities. Previous studies have reported^34^ that Wogonin had strong reversal potency by inhibiting Nrf2 via the reduction of *Nrf2* mRNA at transcriptional processes rather than RNA degradation. Therefore, further studies are necessary undertaken to investigate the mechanism of *Nrf2* mRNA inhibition by Wogonin at transcriptional processes.

## Materials and Methods

### Materials

Wogonin was isolated from S. baicalensis Georgi according to previous protocols^35^. Wogonin was of ≥99% or higher in all experiments, unless otherwise noted. Wogonin was dissolved in dimethyl sulfoxide (DMSO) as a stock solution (100 mM), stored at −20 °C, and diluted to each of the designated concentrations in the buffer solution before each experiment. The final concentration of DMSO did not exceed 0.1%. ADR were purchased from ZheJiang HiSun Pharmacetuical Co., Ltd. (Zhejiang, China). IM was purchased from Melonepharma (Dalian, China). Primary antibodies of β-actin (1:2000), NF-κB (1:500), p-IKKα (1:500), IKKα (1:500), IκBα (1:500) and p-IκBα (1:500) were obtained from Santa Cruz (Santa Cruz, CA). Nrf2 (1:1000), p-ERK (1:1000), Tubulin (1:1000), Stat3 (1:1000), pY705-Stat3 (1:1000) and Lamin A (1:1000) were from Bioworld (OH, USA). RPMI-1640 (Gibico, Carlsbad, CA) and DAPI (Invitrogen, USA) were purchased. The IRDye^TM^ 800 conjugated secondary antibodies were the products of Rockland Inc. (Philadelphia, PA). FITC-conjugated anti-human CD13 antibody was purchased from eBioscience. Epidermal growth factor (EGF) was purchased from Sigma, USA.

### Cell culture and animals

The drug-sensitive human leukemia cell line K562 and its drug-resistant variant K562/A02^36^ and K562R^37^ (IM-resistant K562 cells) were obtained from the Institute of Hematology of Chinese Academy of Medical Sciences (Tianjin, China). The cells were cultured in RPMI 1640 supplemented with 10% fetal bovine serum (Gibco, USA) at 37 °C in 5% CO_2_ in a humidified incubator. The K562/A02 and K562R cells were cultivated in the presence of 1 μg/ml ADR and 0.01 μM IM respectively. Before experiments, ADR and IM were withdrawn from the cells for two generations.

The peripheral blood samples of healthy person (Zhongda Hospital of Southeast University, Nanjing, China) were obtained. Mononuclear cells from the peripheral blood samples were collected using lymphocyte-monocyte separation medium (Jingmei, Nanjing, China). The protocol of collection and of cells complied with guidelines in the Declaration of Helsinki. Mononuclear cells were cultured with RPMI 1640 medium supplemented with 10% FBS. Human monocytes were isolated from mononuclear cells in the attached growth. This study was approved by the responsible Human Participants Ethics Committee of ZhongDa Hospital. All participants were assessed at ZhongDa Hospital and written informed consent was obtained from all of the participants and the methods were carried out in accordance with the approved guidelines.

The animal study was carried out according to the regulations of the State Food and Drug Administration (SFDA) of China on Animal Care. All animal procedures were approved by the Animal Care and Use Committee of the Institute of Biophysics, Chinese Academy of Sciences under the permission number SCXK (SPF2011-0003). NOD/SCID immunodeficient mice (aged 5–6 weeks) were purchased from Shanghai Slac Laboratory Animal Company Limited. The mice were raised in air-conditioned pathogen-free rooms under controlled lighting (12 h light/day) and fed with standard laboratory food and water. K562 cells (K562group) and K562/A02 cells (resistance group) at 2 × 10^6^ were injected into each mouse via tail vein. After one week, the mice inoculated with K562/A02 cells were randomized into four groups (6 mice per group): (1) Untreated group as a negative control; (2) Wogonin monotherapy (40 mg/kg); (3) ADR monotherapy (4 mg/kg); (4) Wogonin combined with ADR. In addition, the mice inoculated with K562 cells were randomized into two groups (6 mice per group): (1) Untreated group as a negative control; (2) ADR monotherapy (4 mg/kg). Wogonin and ADR were given intravenously. Wogonin was given once every other day and ADR was given two times a week. Treatments were as mentioned above. After 30 days, the mice were sacrificed to collect bone marrow, peripheral blood and spleen cells. The leukemia cells were detected by flow cytometry after labeled with FITC-conjugated anti-human CD13 antibody (eBioscience).

### MTT assay

The MTT assay was performed to determine the survival rate of cells incubated with the drugs (1 μg/ml LPS, 40 μM Wogonin) at various times. After treatment for various times, 20 μl MTT dye (5 mg/ml) was added to each well and incubated for an additional 4 h. The dye was solubilized with 100 μl of DMSO, and the plates were read at 570 nm on an automated microtiter plate reader. A blank well that contained only media and drug was used as a control for all the experiments. The inhibitory ratio was calculated using the following formula: inhibitory ratio (%) = (1 − the average absorbance of the treated group/the average absorbance of the control group) × 100%.

### Annexin V/PI staining

K562R cells were harvested after treatment with IM and stained with the Annexin V/PI Cell Apoptosis Detection Kit (KeyGen Biotech, Nanjing, China) according to the manufacturer’s instructions. Data acquisition and analysis were performed with a Becton Dickinson FACS Calibur flow cytometer using Cell-Quest software at Ex./Em.-488/530 nm. The cells in early stages of apoptosis were Annexin V positive and PI negative, whereas the cells in the late stages of apoptosis were both Annexin V and PI positive.

### Western blot analysis

K562/A02 and K562R cells were collected and lysed in lysis buffer (100 mM Tris-HCl, pH 6.8, 4% (m) SDS, 20% (v) glycerol, 200 mM β-mercaptoethanol, 1 mM PMSF, and 1 g/mL aprotinin) for 1 h on ice. The lysates were clarified by centrifugation (13,000 rpm) at 4 °C for 30 min. Protein concentrations in the supernatants were measured using a bicinchoninic acid (BCA) assay kit (Pierce, Rockford, IL, USA) by a Varioskan multimode microplate spectrophotometer (Thermo Waltham, MA, USA). Equal amounts of protein were separated by 8–12% SDS-PAGE. Proteins were detected using specific antibodies, and followed by the IRDyeTM 800 conjugated secondary antibodies for 1 h at 37 °C. Detection was performed using the Odyssey Infrared Imaging System (LI-COR Inc, Lincoln, NE, USA). All blots were stripped and reprobed with polyclonal anti-β-actin or anti-LaminA antibody to ascertain equal protein loadings.

### Real-time quantitative PCR

K562R and K562/A02 cells were pretreated as described above. Total RNA was extracted from cells using the TriPure Isolation Reagent (Roche Diagnostic, Nutley, NJ, USA). Reverse transcription (RT) was performed using equal amounts of mRNA and the quantitative real-time PCR (qPCR) was performed with Takara kit (Takara, Takara BioInc., Otsu, Shiga, Japan); cDNA was collected and saved for real-time quantitative reverse transcription PCR (qRT-PCR). The qPCR assay was performed in a Chromo4TM instrument (BIO-RAD) using the SYBRGreen Master Mix (Applied Biosystems, CA). The relative amount of target mRNA was determined using the comparative threshold (Ct) method by normalizing the target mRNA Ct values to those for β-actin (ΔCt). The sequences of the forward and backward primers of the target genes were as follows: Nrf2, *5*′*-ACACGGTCCACAGCTCATC-3*′and *5*′*-TGTCAATCAAATCCATGTCCTG-3*′; β-actin, *5*′*-TTGCCGACAGGATGCAGAAGGA-3*′ and *5*′*-AGGTGGACAGCGAGGCCAGGAT-3*′.

### Immunofluorescence(IF) confocal microscopy

Treated K562/A02 cells were harvested and seeded onto glass coverslips processed for immunofluorescence. In brief, cells were fixed with 4% paraformaldehyde (PFA) and incubated with Triton X-100. Following the incubation, the cells were blocked with PBS containing 5% BSA for 1 h, and incubated with anti-Nrf2 antibody (1:50) or anti-p65 antibody (1:50) at 37 °C for 1 h. After washing with PBS containing 0.01% Tween 80, the cells were stained with FITC-conjugated anti-rabbit or anti-mouse IgG antibody (1:100) for 1 h. And then the coverslips were stained with DAPI for 30 min. The images were observed under confocal microscopy at 1000× magnification (FV1000; Olympus, Tokyo, Japan).

#### Preparation of cytosolic and nuclear extracts

Cells were harvested in tubes after treatment by ice-cold PBS. Cells were lysed with buffer A (10 mM Hepes-KOH (pH 7.9), 10 mM KCl, 0.1 mM EDTA, 0.5% Nonidet P-40, 1 mM dithiothreitol, 0.5 mM phenylmethylsulfonyl fluoride), incubated on ice for 15 min and then centrifuged. The supernatants were saved as the cytoplasmic fractions. The nuclear pellets were washed three times with buffer A and resuspended of the crude nuclei in high-salt buffer C (20 mM Hepes, 0.5 M KCl, 1 mM EDTA, 1 mM dithiothreitol, 1 mM phenylmethylsulfonyl fluoride, pH 7.9) for 30 min on ice and then centrifuged. The supernatants were collected as the nuclear extracts.

### Electrophoretic mobility shift assays (EMSA)

Nuclear extracts were isolated as described above. According to the manufacturer’s protocol, the experiments with a nonradioactive (biotin label) gel shift assay were performed (Beyotime Institute of Biotechnology, Haimen, China). Briefly, the NF-κB, ARE and Nrf2 oligonucleotide probe was end labeled with biotin with terminal deoxynucleotidyl transferase. Following addition of 5 μl sample buffer, the DNA-protein complexes were resolved on a 6% non-denaturing polyacrylamide gel in a 0.5 × Tris-borate-EDTA buffer at 380 mA for 1 h and then transferred to nylon membrane. Finally, the biotin-labeled DNA was detected by chemiluminescence using the Chemiluminescent EMSA Kit (Beyotime, China) and exposed to X-ray film.

### siRNA transient transfection

The transient transfection assay was carried out in 6-well plates with 3.5 × 10^5^/well K562/A02 or K562R cells in culture medium for 24 h. Then p50siRNA, p65siRNA and Nrf2siRNA were added into the cells with SuperFectinTM II *in vitro* siRNA transfection reagent (Pufei Biotech, ShangHai, China) according to the manufacturer’s instructions, respectively. 50 nM siRNA at final concentration was used in 6-well plates.

### Soft agar colony-formation assay

The experiment was performed when K562/A02 cells were treated with Wogonin and/or ADR for 36 h. Cells were seeded in 6-well plates at 10000/well in 0.8% agar in RPMI-1640 culture medium over a 1.2% agar layer. Subsequently, plates were incubated for 30 days until the colonies were large enough to be visualized. To detect colony size and colony numbers, pictures at 40× magnification were captured by an inverted microscope equipped with a color camera (Nikon Instruments, Inc., Lewisville, TX).

### Promoter assays

To generate the *Nrf2* promoter construct [a], a DNA fragment containing 1.5 kb of the human *Nrf2* promoter region was amplified from genomic DNA with PCR and specific primers: forward, *5*′*-TGGGCGTTGATTGCTATAGTC-3*′, reverse, *5*′*-ATGAGCTGTGGACCGTGTGTT-3*′. The fragment was cloned into the PGL3 basic plasmid (Promega). To generate mutated κB1 (construct [c]) and κB2 (construct [b]) constructs, the PCR primers used were mutκB1 5′-CCAGAGCTGGGAGAAAAACGGTCTACCCAAGAGAACCTCTTCCCAC-3′ and mutκB2 5′-CGCGCGGGCTGAGCTTCCGAACCAACCCCACCCGCG-3′ and. These mutations were introduced with the QuikChange XL Site-Directed Mutagenesis Kit (Agilent). Cells were co-transfected with pNrf2-TA-luc (Sangon Biotech Co., Ltd., Shanghai, China) with Renilla luciferase reporter (as internal control) for 24 h and then treated with or without Wogonin for 24 h. The luciferase activity of cell lysate was detected by the Dual-Luciferase Reporter kit (Promega, Wisconsin, USA) according to the provided protocol. Luciferase signals were collected by Dual Luciferase Assay system (Thermo Fisher Scientific, Rockford, IL).

### Cytokine quantification by enzyme-linked immunosorbent assay

IL-1β secretions in cell supernatants were collected after treatment and measured by the human IL-1β ELISA kits (KeyGEN, Nanjing, China) according to the manufacturer’s instructions. The experiments were repeated three times. Levels of cytokines were expressed in pg/ml.

### Statistical analysis

All results shown represent the mean ± SD from triplicate experiments performed in a parallel manner. Statistical analyses were performed by a one-way ANOVA using the SPSS 11.5 software.

### Ethical approval

All applicable international, national, and/or institutional guidelines for the care and use of animals were followed.

## Results

### NF-κB pathway was involved in the decreased *Nrf2* transcription by Wogonin

To consider the possibility that mutated K-Ras acting through c-Jun and c-myc activation via Raf/MEK/ERK pathway might lead to an increase in *Nrf2* transcription, as recently shown in pancreatic cancer^38^, we sought to determine whether the MEK activator EGF could reverse the inhibitory effect of Wogonin on the expression of *Nrf2* mRNA in K562/A02 and K562R cells. However, in K562/A02 cells, EGF had no effect on Wogonin-mediated *Nrf2* mRNA expression (Fig. 1A) despite significantly inducing p-ERK at 10 μM at 2 and 4 hours after treatment (Fig. 1C and E). Similarly, EGF had no effect on Wogonin-mediated inhibition of *Nrf2* mRNA expression in K562R cells (Fig. 1B) in despite of inducing p-ERK (Fig. 1D and E). Together with the fact that K-Ras mutations were rare in CML (circa 5% of CML), the findings suggested that this pathway was not responsible for the decreasing *Nrf2* transcription by Wogonin.

Recent studies reported NF-κB activation contributed to high expression of Nrf2 and an inhibitor of IκB phosphorylation (BAY11-7082) reduced *Nrf2* mRNA expression in AML^19^. Therefore, we investigated whether Wogonin-mediated inhibition of *Nrf2* mRNA was dependent on downregulation of NF-κB signaling. As Fig. 1F and G indicated the ratio of p-IκBα/IκBα and p-IKKα/IKKα expression was high in K562/A02 cells and K562R cells (also in Supplementary Fig. 1A and B). However, when resistant cells were incubated with Wogonin, phosphorylation of IκBα and IKKα expression were both suppressed significantly in a concentration-dependent manner (as Fig. 1F and G indicated). Moreover, p65 was reduced by Wogonin in the nucleus of resistant CML cells, and the analysis showed reduction of both Nrf2 and p65 nuclear protein levels to correlate in a 1:1 manner (Fig. 2A and B, also in Supplementary Fig. 2A and B).

To further understand the involvement of NF-κB pathway in Wogonin mediated-*Nrf2* mRNA regulation in K562 resistant cells, we used an activator of NF-κB, LPS. As shown in Fig. 2C and D, after treatment with 1 μg/ml LPS for 4 h, K562 resistant cells exhibited increased *Nrf2* mRNA expression. However, LPS significantly blocked the inhibitory effect of Wogonin on the expression of *Nrf2* mRNA (Fig. 2C and D). Additionally, IF analysis showed that Wogonin significantly suppressed NF-κB and Nrf2 nuclear translocation in K562/A02 cells (Fig. 2E), while the inhibition of Wogonin-mediated Nrf2 nuclear translocation was blocked by treatment with LPS (Fig. 2E). These results illustrated that inhibition of NF-κB pathway played an important role in downregulation of *Nrf2* mRNA expression by Wogonin.

### Inhibition of the κB activity is responsible for reducing *Nrf2* transcription by Wogonin

Analysis with EMSA using nuclear extracts from treated cells showed (also in Supplementary Fig. 3A and B): compared with untreated cells (Fig. 3A and B, lane 6), Wogonin and BAY11-7082 inhibited the recruitment of Nrf2 to ARE in K562/A02 cells and K562R cells as indicated in lane 8 and 10, respectively. Treatment with LPS in K562/A02 cells and K562R cells increased the binding of Nrf2 to ARE as indicated in lane 7. However, the inhibition of the binding of Nrf2 to ARE sites was reversed by treatment with LPS (Fig. 3A and B) as indicated in lane 9. Additionally, we also observed a retarded supershift band in the presence of an anti-Nrf2 antibody, further indicating the presence of Nrf2 in the complex (anti-Nrf2 antibody + Nrf2 + biotin-ARE sequence; Fig. 3A and B, lane 5). To further clarify the role of the NF-κB subunits p50 and p65 in the regulation of Wogonin-mediated Nrf2 reduction in K562/A02 cells, we used siRNA knockdown to silence p50 and p65. siRNA constructs, effective at silencing p50 or p65 (Fig. 3C and D-left, also in Supplementary Fig. 4A and B), individually and in combination were also able to inhibit the binding of p50 and p65 to the κB sites of K562 resistant cells in a κB-binding assay (Fig. 3C and D-right). In control K562 resistant cells, Fig. 3E and F showed an increase of *Nrf2* mRNA in response to LPS, and a decrease in *Nrf2* mRNA when treated with BAY11-7082. Wogonin was also able to effectively inhibit *Nrf2* mRNA levels. By contrast, treatment with LPS significantly reduced the inhibition of Wogonin- mediated *Nrf2* mRNA. Importantly, there was no effect on the inhibition of *Nrf2* mRNA by Wogonin at silencing p50 or p65, individually and in combination (Fig. 3E and F). The findings indicated that Wogonin inhibited the κB-binding activity, resulting in *Nrf2* mRNA downregulation in K562 resistant cells. NF-κB is a key regulator of pro-inflammatory cytokine IL-1β, therefore we investigated the effect of Wogonin on the secretion of IL-1β in K562/A02 and K562R cells. As expected, ELISA revealed that Wogonin substantially decreased IL-1β secretion in a concentration-dependent manner compared with untreated cells (Fig. 4A and B). Thus, Wogonin inhibited NF-κB signaling pathway which was further confirmed by reduction of IL-1β secretion.

### Understanding the regulation of Nrf2 by Wogonin via κB2 inhibition

To determine the role of the κB-binding sites within the *Nrf2* promoter sequence in regulating Nrf2 by Wogonin in K562 resistant cells, we created κB-deletion mutant reporter constructs of the human *Nrf2* promoter (Fig. 4C). K562/A02 cells and K562R cells were transfected with each individual construct and assayed in the presence of NF-κB inhibition (BAY11-7082) and NF-κB activation (LPS) with or without Wogonin. The mutated κB2 construct [b] showed decreased basal levels of promoter activity compared with wild-type *Nrf2* promoter construct (Fig. 4D and E). However, the mutated κB1 construct [c] showed similar promoter activity to those seen with the wild-type *Nrf2* promoter construct (Fig. 4D and E). As a positive control we treated transfected cells with LPS and BAY11-7082 alone. Figure 4D and E showed an increase in promoter activity in wild-type *Nrf2* promoter construct [a] and the mutated κB1 construct [c] but not mutated κB2 construct [b] in response to LPS, and a decrease in promoter activity in wild-type *Nrf2* promoter construct [a] and the mutated κB1 construct [c] but not mutated κB2 when treated with BAY11-7082. In the wild-type *Nrf2* promoter construct, Wogonin was also able to effectively inhibit the *Nrf2* promoter activity. By contrast, treatment with LPS significantly reduced the inhibition of Wogonin-mediated *Nrf2* promoter activity. Moreover, the construct with mutated κB1 showed similar promoter activity to those seen with the wild-type *Nrf2* promoter construct (Fig. 4D and E). However, the construct with mutated κB2 showed no effect on Wogonin-mediated *Nrf2* promoter activity after treatment with LPS. Further analysis with EMSA using nuclear extracts showed that Nrf2 probe in cold competition including mutated κB2 regions no κB1 regions did not suppress the binding of NF-κB subunit p65 to *Nrf2* sequence (Fig. 4F). However, wild-type *Nrf2* probe including normal κB2 regions no κB1 regions could suppress NF-κB binding activity. Figure 4F showed Wogonin decreased the Nrf2 binding activity in biotin-Nrf2 probe including κB2 regions alone, and LPS could reverse the decreased binding activity in response to the combination of Wogonin and LPS. These results demonstrated the κB2 site, located at +270 upstream of the transcription start site, was responsible for the decreased expression of Nrf2 by Wogonin in resistant CML cells.

### Downregulation of pY705-Stat3 contributed to inhibition of the NF-κB binding by Wogonin

Recent emerging reports demonstrated Stat3 was required to maintain tumor NF-kB activity^39^. Therefore, we investigated whether Wogonin-mediated NF-κB inactivation was dependent on downregulation of pY705-Stat3. High constitutive levels of pY705-Stat3 were observed and independent on BCR/ABL in resistant CML cells (Fig. 5A). In fact, IM completely dephosphorylated BCR/ABL, indicating that IM resistance was BCR/ABL independent in resistant CML cells. However, as Fig. 5A showed, when K562/A02 cells were incubated with different concentrations of Wogonin, expression of pY705-Stat3 was decreased significantly in a concentration-dependent manner, but p-BCR/ABL expression was not affected. These date suggested that downregulation of Stat3 phosphorylation on tyrosine 705 by Wogonin did not rely on p-BCR/ABL levels. To further explore whether inhibition of Stat3 activity contributed to Wogonin-mediated NF-κB inactivation, Stat3 was overexpressed in resistant CML cells. As shown in Fig. 5B, p65 nuclear translocation was restored by ectopic Stat3 in the presence of Wogonin, which was likely due to the interruption of Stat3-mediated crosstalk between Wogonin and NF-κB inactivation. To further ascertain the relationship between Stat3 and NF-κB inhibition in the presence of Wogonin, we examined NF-κB activity by EMSA. As illustrated in Fig. 5C, data showed Wogonin significantly reduced the effective binding of p65 to the biotin-labeled oligonucleotide Nrf2 probe (including κB2 site). However, after transfection of Stat3 plasmid, the reduction of the binding of p65 to κB2 by Wogonin was reversed (Fig. 5C). Above all, these results illustrated that Wogonin suppressed the binding of p65 to Nrf2 at κB2 site by inhibition of pY705-Stat3, which was independent on BCR/ABL.

### Wogonin enhanced chemotherapy-induced apoptosis via inhibition of Nrf2

To investigate whether apoptosis induced by chemotherapy could be enhanced by Wogonin, AnnexinV/PI staining assay was performed. Apoptosis phenomenon was exhibited more markedly when treatment with Wogonin and IM together compared with IM alone in K562R cells. As shown in Fig. 6A, 0.5 μM IM treatment for 24 h resulted in apoptosis of K562R cells by 14.89%. Compared with IM treatment alone when 0.5 μM IM was combined with 10, 20 and 40 μM Wogonin, the mean apoptotic population of K562R cells increased 1.9-fold (28.14 ± 4.32%), 3.2-fold (47.04 ± 3.51%), and 5.6-fold (82.94 ± 2.36%) respectively, including both the early and the late apoptotic cells. And there was no significant apoptosis in 10, 20, and 40 μM of Wogonin^34^. Moreover, Nrf2 knockdown resulted in no significant reduction in the actual number of colonies that were formed (Fig. 6B). However, the addition of ADR showed that Nrf2 knockdown resulted in a significantly augmented chemotherapy-induced reduction in colony formation in the high-Nrf2 expressing resistant CML cells (Fig. 6B). The combination of ADR with Wogonin markedly decreased the number of colony formation in resistant K562/A02 cells (Fig. 6B). If the promoter of *Nrf2* did contain an authentic κB binding site and CML cells did not have genetic aberrance in the Nrf2 pathway, then activation of the NF-κB pathway would enhance *Nrf2* mRNA in normal cells. We have shown that LPS could induce *Nrf2* mRNA in THP-1 cells by up to 4-fold (Fig. 6C). To determine whether Wogonin down-regulated *Nrf2* mRNA by NF-κB signaling in other cells, we stimulated human monocytes and THP-1 cells by LPS with and without BAY11-7082 treatment. Data demonstrated that LPS induced *Nrf2* mRNA in human monocytes cells, and Wogonin reduced the up-regulation of *Nrf2* mRNA by LPS (Fig. 6C). LPS-induced *Nrf2* mRNA was almost reverted back to normal by BAY11-7082 treatment (Fig. 6C). Meanwhile, IL-1β secretion was stimulated by LPS and inhibited by Wogonin with and without BAY 11-7082 treatment in normal cells and THP-1 cells (Fig. 6D). Thus, the results revealed Wogonin also reduced the induced expression of *Nrf2* mRNA in normal monocyte cells.

### Wogonin potentiated the inhibitory effect of ADR on leukemia development *in vivo*

#### Wogonin potentiated the inhibitory effect of ADR on tumor growth in NOD/SCID mice

The study *in vivo* aimed to examine the effect of ADR combining with Wogonin and was performed by xenografted model. We transplanted K562 cells and K562/A02 cells into NOD/SCID mice by intravenous injection. 7 days later, >1% CD13^+^ cells were detected in mice peripheral blood, indicating that numerous human K562 and K562/A02 cells had engrafted and proliferated in the experimental animals. Then the animals transplanted K562/A02 cells were treated with or without ADR (4 mg/kg), together with or without Wogonin (40 mg/kg), and the animals transplanted K562 cells were treated with or without ADR. For the duration of treatment (30 days) all tested mice were alive. 4 weeks later, the blood routine examination was monitored when all mice was killed. At the indicated concentration of Wogonin, there was no significantly toxicity. The expression of the significant surface antigen CD13^+^ on K562 and K562/A02 cells was analyzed by FACS. As shown in Fig. 7A, a substantial reduction in CD13^+^ cells in BM cells obtained from combination group was observed. The data of the non-treated group was 14.57 × 10^6^/ml and the combined group was 7.47 × 10^6^/ml. There was also significantly reduction in CD13^+^ cells of spleen and PB in the combination group compared with non-treated K562/A02 group. The results with combined treatment in transplanted K562/A02 cells were similar with the ADR treatment in transplanted K562 cells (Fig. 7A). Organs (spleen and liver) were excised from the animals and weighed. Livers (Fig. 7B) and spleens (Fig. 7C) of group treated with agents in combination recovered the weight of normal spleens and livers. Histological evaluation of the tissues revealed marked leukemia cell infiltration of the spleen and liver. Spleen of control group showed normal histology with splenic parenchyma composed of normal white pulp and red pulp and a normal splenic capsule and trabeculae. As shown in Fig. 7D, leukemia induced group and Wogonin treated group exhibited effacement of architecture of the spleen with prominent extramedullary hematopoiesis comprising of infiltration by myeloid cells and numerous megakaryocytes as well as infiltration by neoplastic cells with large nuclei and scanty cytoplasm. Administration with ADR in combination with Wogonin restored the normal architecture of the spleen. The liver of control group was composed of cords of normal hepatocytes with intervening sinusoids. Normal portal tracts and central veins were seen. In Wogonin treated group and leukemia induced group, the liver showed infiltration by neoplastic cells and multiple foci of extramedullary hematopoiesis (Fig. 7D). Subsequent to treatment with ADR combined with Wogonin, the histology of liver reverted back to normal.

#### Wogonin combined with ADR treatment against leukemic cells by suppressing NF-κB/Nrf2 pathway *in vivo*

To address the potential mechanism of Wogonin in combination with ADR against leukemic cells *in vivo*, Western blot and immunohistochemistry were performed. Western blot results of leukemic cells revealed that up-regulation of Nrf2 and p65 as well as p-Stat3 translocated into nuclei in untreated K562/A02 group (Fig. 8A). But mice treated with ADR and Wogonin in combination had reduced nuclear NF-κB p65, p-Stat3 and Nrf2 expression (Fig. 8A). We also found that Wogonin suppressed phosphorylation of IKKα and IκBα (Fig. 8B). *Nrf2* mRNA expression was significantly reduced by Wogonin monotherapy group and the combination group in K562/A02 group (Fig. 8C). RT-PCR revealed that mice treated with ADR and Wogonin in combination had reduced IL-1β mRNA expression in the peripheral blood (Fig. 8D). Spleen were excised and analyzed by using immunohistochemical staining. As illustrated in Fig. 8E, NF-κB p65 and Nrf2 expression were increased in spleen in untreated K562/A02 group, but Wogonin reduced NF-κB p65 and Nrf2 expression in spleen.

## Discussion

Wogonin-mediated inhibition of Nrf2 was not linked to up-regulation within Keap1, but was in fact the result of down-regulation of *Nrf2* mRNA through posttranscriptional regulation in resistant CML cells^34^. However, less is known about the precise mechanism of the transcriptional regulation of Nrf2 by Wogonin in resistant cells. In this study, we found a directly functional correlation between downregulation of *Nrf2* mRNA and NF-κB transcription factors *in vitro* and *in vivo*. Furthermore, p-Stat3 reduction was found to be involved in NF-κB inactivation by Wogonin. Pretreatment with LPS, significantly reversed the inhibitory effect of Wogonin on the expression of Nrf2 and *Nrf2* mRNA. *In vivo*, Histological evaluation of the tissues revealed Wogonin combined with ADR attenuated marked leukemia cell infiltration of the spleen and liver. Moreover, Western blot and immunohistochemistry revealed that the animals treated with Wogonin significantly suppressed pY705-Stat3 and Nrf2 signaling.

It is now becoming recognized that many transcription factors control the expression of the Nrf2 gene. Among the transcription factors, NF-κB and AP-1 families are arguably the most important, and the best studied regulators of the cellular stress response in vertebrates^40^. In this study, we firstly investigated Wogonin significantly decreased the ratio of p-IκBα/IκBα and p-IKKα/IKKα expression in a concentration-dependent manner. Moreover, Western blot analysis and immunofluorescence staining showed that Wogonin markedly suppressed NF-κB nuclear translocation in K562/A02 and K562R cells. We further found that the inhibitory effect of Wogonin on the expression of Nrf2 and *Nrf2* mRNA was reversed by LPS in resistant cells, which was analyzed by RT-PCR and IF. These data indicated that inhibition of NF-κB signaling played an important role in downregulation of *Nrf2* mRNA expression by Wogonin in the reversal experiments. Several studies have indicated that NF-κB pathway could control the induced expression of Nrf2 in normal cells, as well as cancer cells, under the stimulation of LPS^41^. However, a research article reported^42^ that high concentrations of Wogonin inhibited NF-κB signaling pathway and induced activation of Nrf2 signaling pathway in inflammation-associated colon carcinogenesis. The opposite actions of Wogonin on the Nrf2 signaling pathway might be due to a different Nrf2 function in response to different concentrations of Wogonin and cell-type specific. Thus, we assumed that this discrepancy of Wogonin on Nrf2 signaling pathway between resistant tumors and inflammation-associated colon carcinogenesis is the result of completely different machinery. Other transcription factors, including heat shock factors, signal transducers and activators of transcription proteins, hypoxia-inducible factor-1, CCAAT/enhancer binding protein factors, and USF family members^43^, are known to regulate HO-1 transcription under specific circumstances and may work in conjunction with Nrf2.

Recent emerging reports demonstrated that the Nrf2 pathway acted as a double-edged sword: it protected the body from chemical carcinogenesis and environmental stresses but provided advantages for the growth and development of cancer cells^44^. Many studies in the field have focused on identification of activation of Nrf2 as ‘bad’ for cancer patients during the course of chemotherapy^45^, as evidenced by our finding that modulation of the Nrf2-mediated response affected the resistant carcinogenic process in response to chemotherapeutic agents. Low concentrations of Wogonin (10–40 μM) with safety and low-toxicities showed the strong potency to increase chemotherapeutic agents induced apoptosis though inactivation of Nrf2 via NF-κB signaling in the resistant cancer cells.

Wogonin-mediated activity of Nrf2/ARE pathway was inhibited primarily through posttranscriptional regulation. Our current findings by EMSA showed that NF-κB activation by LPS blocked Wogonin-mediated reduction of the binding of Nrf2 to ARE. To further clarify the role of NF-κB subunits in the transcriptional regulation of Nrf2 by Wogonin, p65 siRNA and p50siRNA or the combination were used. Here, it is worth reminding that both p65 and p50 played a key role in reduction of *Nrf2* mRNA induced by Wogonin. Collectively, these findings implicated that inhibition of the binding activity of κB was involved in Wogonin-mediated reduction of *Nrf2* mRNA. As expected, when the binding activity of κB disappeared by silencing p65 and p50, the level of *Nrf2* mRNA was not changed in response to Wogonin or NF-κB activation and inhibition. Small molecules and viral vectors that inhibit IKK, or other aspects of the NF-κB activation pathways, have been shown to induce cell death and inhibit the proliferation of tumors or tumor-derived cell lines^46^. The concept that inhibition of NF-κB suppressed *Nrf2* transcription was consistent with NF-κB classic role in stimulating the transcription of target genes. Meanwhile, several recent studies have supported the theory that inhibition of NF-κB by natural drugs might downregulate cellular responses to specific stimuli. For example, Gambogic acid inhibited CDDP-induced upregulation of the Nrf2-HO-1 pathway through inactivation of NF-κB signaling^47^. In addition, Liu *et al*.^48^ reported that the elevated HO-1 of Nrf2 downstream gene was associated with increased activity of the nuclear NF-κB and the inhibition of NF-κB led to the block of its induction. However, the specific mechanism of NF-κB inhibition by natural drugs involving in downregulation of cellular responses was not previously described in any other tumor type. Several studies have indicated that the human *Nrf2* promoter contained several transcription factor-binding sites, including two κB-binding sites located downstream of the ARE^49^. To determine if any of these sites were important in the down-regulation of Nrf2 by Wogonin in resistant CML cells, we created site-directed mutants of the human *Nrf2* promoter, which removed one or the other of the κB sites. Interestingly, the construct with mutated κB2 showed no effect on the reduced *Nrf2* promoter activity after treatment with Wogonin or NF-κB activation and inhibition. However, the construct with mutated κB1 showed treatment with LPS significantly reversed the inhibition of Wogonin-mediated *Nrf2* promoter activity, which was similar promoter activity to those seen with the wild-type *Nrf2* promoter construct. Hence, these results indicated that the κB2 site, located at +270 upstream of the transcription start site, was responsible for the decreased expression of Nrf2 by Wogonin in resistant CML cells.

Crosstalk between Stat3 and NF-kB has been demonstrated at multiple levels, including activation of Stat3 by NF-kB-regulated factors such as IL-6^50^. A recent study reported that Stat3 interaction with p65 led to overexpression of the immunosuppressive IL-23/p19 gene^51^. NF-kB activity regulating multiple critical oncogenic processes was determined in part by its interaction with activated Stat3. However, Wogonin had an inhibitory effect on those pathways in resistant CML cells. If the promoter of Nrf2 did contain an authentic κB binding site and CML cells did not have genetic aberrance in the Nrf2 pathway, then activation of the NF-κB pathway would enhance *Nrf2* mRNA in normal human monocytes. Therefore, we stimulated human monocytes and THP-1 cells with LPS for the next experiments. Data demonstrated that LPS induced *Nrf2* mRNA in human monocytes cells, and Wogonin reduced *Nrf2* mRNA by NF-κB signaling. However, several dietary antioxidants and NF-κB inhibitors, including MG132, PDTC, curcumin, and a-lipoic acid, have all been shown to induce HO-1 through Nrf2 activation. One possible explanation for these observations was the mechanism by which NF-κB significantly regulated varies in different cell subtypes. Interestingly, a previous finding also observed that p50 (and to a lesser extent p65) could bind to the ARE site at −4100^22^. How p50 interacts with the ARE by Wogonin is unknown. Hence, our future studies will determine the interplay between p50, Nrf2, and ARE in the presence of Wogonin stimuli. This was not the first time that another transcription factor has been associated with Nrf2 and the ARE-binding site. For example, a recent study showed that p53 suppressed Nrf2-dependent transcription by displacing Nrf2 bound to the promoter of ARE-dependent genes^52^. Further work to delineate which mechanism of NF-κB inactivation by Wogonin for inhibition of transcription of *Nrf2* offers the possibility of paving the way for the development of combination therapies more effective in the treatment of CML.

As shown in Fig. 9, Wogonin suppressed the activity of Nrf2/ARE pathway in resistant CML cells at posttranscriptional regulation via NF-κB inactivation. Furthermore, the NF-κB subunits p50 and p65 seemed to be responsible for this suppression of *Nrf2* transcription by binding to only one of the κB sites in the *Nrf2* promoter. The following findings confirmed the κB2 site was responsible for the decreased expression of Nrf2 by Wogonin in resistant K562 cells. Moreover, reduction of p-Stat3 was found to be involved in Wogonin-mediated inhibition of the κB2 binding activity. *In vivo*, Western blot and immunohistochemistry revealed that the animals treated with Wogonin monotherapy or in combination significantly suppressed p-Stat3 and Nrf2. Therefore, identification of Wogonin is a potent small-molecule inhibitor of Nrf2/ARE pathway, and developing it into druggable compounds may be used to increase the efficacy of anticancer drugs or reverse drug resistance during chemotherapy. Thus, further studies in other animal models as well as in human clinical trials are necessary to test the efficacy of co-administration of Wogonin as well as other Nrf2 inhibitors during the prevention and treatment of cancer.

## Additional Information

**How to cite this article**: Xu, X. *et al*. Wogonin reversed resistant human myelogenous leukemia cells via inhibiting Nrf2 signaling by Stat3/NF-κB inactivation. *Sci. Rep.* **7**, 39950; doi: 10.1038/srep39950 (2017).

**Publisher's note:** Springer Nature remains neutral with regard to jurisdictional claims in published maps and institutional affiliations.

## Supplementary Material

Supplementary Information

## Figures and Tables

**Figure 1:** Wogonin decreased p-IKKα and p-IκBα. (**A**,**B**) K562/A02 and K562R cells were pretreated with 50ng/ml EGF for 4 h and then treated with or without 40 μM Wogonin for 24 h. Levels of *Nrf2* mRNA in treated K562, K562/A02 and K562R cells were determined by RT-PCR. *p < 0.05 versus untreated K562 cells. ^#^p < 0.05 versus untreated K562/A02 or K562R cells. (**C,D**) K562/A02 and K562R cells were treated with 50ng/ml EGF for 2 h and 4 h. The expression of the downstream gene p-ERK was detected by Western blot in treated cells. (**E**) The expression of p-ERK was analyzed at 2 h and 4 h after treatment with 50ng/ml EGF. *p < 0.05 versus untreated K562/A02 or K562R cells. (**F**,**G**) K562/A02 and K562R cells were exposed to various concentrations of Wogonin (10, 20, and 40 μM) for 24 h. p-IkBα/IkBα and p-IKKα/IKKα was analyzed by Western blot analysis. *p < 0.05 versus untreated K562 cells. ^#^p < 0.05 versus untreated K562/A02 or K562R cells. All results were represented as the mean ± SD of three independent experiments.

**Figure 2:** Wogonin inhibited Nrf2 transcription via NF-κB pathway. (**A**,**B**) The expression of nuclear protein p65 and Nrf2 was assessed by Western blot analysis in treatment with 5 μM BAY11-7082 for 6 h or various concentrations of Wogonin for 24 h in K562/A02 and K562R cells, respectively. Nuclear protein expression was normalized to lamin A levels. *p < 0.05 versus untreated cells. (**C**,**D**) K562/A02 and K562R cells were pretreated with 1 μg/ml LPS for 4 h and then treated with or without 40 μM Wogonin for 24 h. Levels of *Nrf2* mRNA in treated K562, K562/A02 and K562R cells were determined by RT-PCR. *p < 0.05 versus untreated K562 cells. ^#^p < 0.05 versus untreated K562/A02 or K562R cells. ^a^p < 0.05 versus 40 μM Wogonin. (**E**) K562/A02 cells were pretreated with 1 μg/ml LPS for 4 h and then treated with or without 40 μM Wogonin for 24 h, respectively. Nuclear translocalization of p65 and Nrf2 was assessed by IF using a confocal laser microscope, Nrf2 (green), p65 (red), DAPI (blue). All results were represented as the mean ± SD of three independent experiments.

**Figure 3:** Inhibition of the κB activity was responsible for reducing Nrf2 transcription by Wogonin. (**A**,**B**) 40 μM Wogonin and 5 μM BAY11-7082 reduced the binding of Nrf2 to ARE, respectively. However, the inhibition of the binding of Nrf2 to ARE sites was reversed by treatment with 1 μg/ml LPS. Nrf2/ARE DNA binding activity was assessed by EMSA after treatment with 40 μM Wogonin or BAY11-7082 in the presence or absence of LPS. (**C**,**D**) Left: Cells were treated by silencing p50 or p65, individually and in combination, and then the level of p50 and p65 was detected by Western blot analysis in K562/A02 and K562R cells. Right: After cells transfected with the indicated siRNAs, NF-κB DNA binding activity was assessed by EMSA. (**E**,**F**) K562/A02 and K562R cells were transiently transfected with indicated siRNAs shown in each plot and controlsiRNA for normalization of transfection efficiency. Cell extracts were harvested, and the level of *Nrf2* mRNA was determined by RT-PCR. LPS (1 μg/ml) treatment acted as a positive control to activate NF-κB and BAY 11-7082 (5 μM) to inhibit NF-κB. *p < 0.05 versus transfected with controlsiRNA in untreated cells. ^#^p < 0.05 versus untreated controls. All results were represented as the mean ± SD of three independent experiments.

**Figure 4:** Understanding the regulation of Nrf2 by Wogonin via κB2. (**A**,**B**) K562/A02 and K562R cells were treated with various concentrations of Wogonin, and IL-1β secretion was determined by ELISA. *p < 0.05 versus control. (**C**) Schematic presentation of the Nrf2 promoter constructs that were created for this study, being either wild-type [a], κB2 site-deleted [b], or κB1 site-deleted [c], constructs. (**D**,**E**) K562/A02 and K562R cells were transiently transfected with each promoter construct and PGL3 for normalization of transfection efficiency. The supernatant extracts in lysis buffer were harvested, and detected by luciferase assays. *p < 0.05 versus transfected with untreated Nrf2 wild-type control. ^#^p < 0.05 versus untreated controls. LPS (1 μg/ml) treatment acted as a positive control to activate NF-κB and BAY 11-7082 (5 μM) to inhibit NF-κB. (**F**) The binding of NF-κB subunit p65 to Nrf2 sequence was assessed by EMSA after treatment. Wogonin decreased the p65 binding activity in biotin-Nrf2 probe including κB2 regions alone, and LPS could reverse it. Cold competition probe including mutated κB2 regions no κB1 regions and wild-type Nrf2 probe including normal κB2 regions no κB1 regions. All results were represented as the mean ± SD of three independent experiments.

**Figure 5:** Downregulation of pY705-Stat3 was responsible for inhibition of the p65 binding activity by Wogonin. (**A**) After treatment with or without 40 μM Wogonin for 24 h, the expression of pY705-Stat3, p-BCR-ABL and Stat3 were examined by Western blot assays in K562/A02 cells. *p < 0.05 versus untreated K562/A02 cells. (**B**) Transfected K562/A02 cells with Stat3 plasmid were exposured to 40 μM Wogonin for 24 h, pY705-Stat3 and p65 were examined by Western blot. *p < 0.05 versus untreated K562/A02 cells. (**C**) The binding of NF-κB subunit p65 to Nrf2 sequence including κB2 site was assessed by EMSA after treatment. K562/A02 cells were transfected with Stat3 plasmid and then exposured to 40 μM Wogonin. Cell nuclear extracts were analyzed. Wogonin decreased the p65 binding activity in biotin-Nrf2 probe including κB2 regions alone, and Stat3 plasmid could reverse it. *p < 0.05 versus control. All results were represented as the mean ± SD of three independent experiments.

**Figure 6:** Wogonin enhanced chemotherapy-induced apoptosis via inhibition of Nrf2. (**A**) K562R cells were treated with or without 0.5 μM IM in the absence or presence of Wogonin for 24 h, respectively. Annexin V/PI double-staining assay of treated K562/A02 cells was analyzed by flow cytometry. *p < 0.05 versus treatment with IM. (**B**) Soft-sugar-colony forming experiment was performed to ascertain Wogonin reversal effect by Nrf2 signaling. *p < 0.05 and **p < 0.01 versus control. (**C**) Human monocytes and THP-1 cells were treated with LPS in the absence or presence of BAY11-7082 and Wogonin. Levels of Nrf2mRNA in treated cells were determined by RT-PCR. *p < 0.05 versus control. ^#^p < 0.05 and ^##^p < 0.01versus LPS (1 μg/ml). (**D**) Human monocytes and THP-1 cells with LPS in the absence or presence of BAY11-7082 and Wogonin. IL-1β secretion was determined by ELISA after treatment. *p < 0.05 versus control. ^#^p < 0.05 versus LPS (1 μg/ml). All results were represented as the mean ± SD of three independent experiments.

**Figure 7:** Wogonin potentiated the inhibitory effect of ADR on tumor growth in NOD/SCID mice. Tumor xenografts inoculated with K562 and K562/A02 cells (resistance group). Then the transplanted animals were treated with ADR (4 mg/kg) by intravenous injection two times a week; Wogonin (40 mg/kg) intravenous injection was performed every other day for 4 weeks. (**A**) CD13^+^ cells of BM, PB and spleen were detected by flow cytometry. *p < 0.05 versus untreated K562 group. ^#^p < 0.05 compared with untreated K562/A02 group. (**B**,**C**) The weight of livers and spleens was analysis. *p < 0.05 versus untreated K562 group. ^#^p < 0.05 compared with untreated K562/A02 group. (**D**) The spleens and livers were examined for H&E staining. All results were represented as the mean ± SD of three independent experiments.

**Figure 8:** Wogonin combined with ADR treatment against leukemic cells by suppressing Stat3/Nrf2 pathway *in vivo*. (**A**) The expression of nuclear protein pY705-Stat3, p65 and Nrf2 were examined by Western blot assays in leukemic cells. *p < 0.05 compared with control. ^#^p < 0.05 compared with K562/A02 group. (**B**) The ratio of p-IkBα/IkBα and p-IKKα/IKKα was analyzed by Western blot in leukemic cells. *p < 0.05 compared with control. (**C**) Levels of *Nrf2* mRNA in untreated or treated group in leukemic cells were determined by RT-PCR. *p < 0.05 compared with control. ^#^p < 0.05 compared with K562/A02 group. (**D**) Levels of IL-1βmRNA in untreated or treated group were determined by RT-PCR. *p < 0.05 compared with control. ^#^p < 0.05 compared with K562/A02 group. (**E**) Nuclear NF-κB p65 and Nrf2 expression in spleen were analyzed by using immunohistochemical staining. All results were represented as the mean ± SD of three independent experiments.

**Figure 9:** Schematic representation of the molecular mechanisms proposed in the reversal effect of Wogonin via inhibition of p-Stat3/κB2/Nrf2 in resistant CML cells.
